The article "Implementing Multilabeling, ADASYN, and ReliefF Techniques for Classification of Breast Cancer Diagnostic through Machine Learning: Efficient Computer-Aided Diagnostic System" was published in 2021. Journal: J Healthc Eng.

# Implementing Multilabeling, ADASYN, and ReliefF Techniques for Classification of Breast Cancer Diagnostic through Machine Learning: Efficient Computer-Aided Diagnostic System

**DOI:** 10.1155/2021/5577636

**Published:** 2021-03-22

**Authors:** Taha Muthar Khan, Shengjun Xu, Zullatun Gull Khan, Muhammad Uzair chishti

**Affiliations:** ^1^Department of Control Science and Engineering, Xi'an University of Architecture and Technology, Xi'an, Shaanxi 710055, China; ^2^Department of Computer Science, Air University, Islamabad, Pakistan; ^3^Department of Computer Science, National Collage of Business Administration Lahore Sub-Campus, Multan, Pakistan

## Abstract

Multilabel recognition of morphological images and detection of cancerous areas are difficult to locate in the scenario of the image redundancy and less resolution. Cancerous tissues are incredibly tiny in various scenarios. Therefore, for automatic classification, the characteristics of cancer patches in the X-ray image are of critical importance. Due to the slight variation between the textures, using just one feature or using a few features contributes to inaccurate classification outcomes. The present study focuses on five different algorithms for extracting features that can extract further different features. The algorithms are GLCM, LBGLCM, LBP, GLRLM, and SFTA from 8 image groups, and then, the extracted feature spaces are combined. The dataset used for classification is most probably imbalanced. Additionally, another focal point is to eradicate the unbalanced data problem by creating more samples using the ADASYN algorithm so that the error rate is minimized and the accuracy is increased. By using the ReliefF algorithm, it skips less contributing features that relieve the burden on the process. Finally, the feedforward neural network is used for the classification of data. The proposed method showed 99.5% micro, 99.5% macro, 0.5% misclassification, 99.5% recall rats, specificity 99.4%, precision 99.5%, and accuracy 99.5%, showing its robustness in these results. To assess the feasibility of the new system, the INbreast database was used.

## 1. Introduction

Breast cancer is considered a key health issue in women which is causing a high rate of casualty. The initial diagnosis of breast cancer with mammographic screening and appropriate pharmacological treatments has steadily increased the prognosis of breast cancer [1]. These include mammography, biopsy, ultrasound image, and thermography [2]. The biopsy is painful procedure and rather expensive. Chemotherapy is usually frailty associated with a psychiatric condition defined as the accumulation of several interactive diseases, impairs, and disability: exhaustion, nausea, inadequate, relatively slow walking speed and physical exercise, and unintended weight loss [3, 4]. So, some doctors recommended dispensing low-dose aspirin before and after the detection of breast cancer [5]. But today's world image recognition methods have an important role to play in the analysis of tumor images by using a machine learning methodology. It uses a random generator, a function extractor, and a classifier to model a doctor's enquiry and construct a personalized questionnaire [6]. Also microwave-based imaging techniques were developed for breast cancer detection [7]. The data mining as well as classification techniques is a well-organized approach of classifying data. Particularly in the medical field, these approaches are commonly useable diagnostics research for decision making. Many classification methods are used in the algorithms of machine learning like decision tree (C45), support vector machine (SVM), and naive Bayes algorithm [8]. Support vector machine (SVM) discriminatory classifier is used to classify hyperplanes for binary groups. But, in particular case, the major drawback is low results for a greater number of characteristics than the number of samples [9]. The decision tree (C4.5) is a hierarchical decision support technique, but its downside is that it is highly unreliable and data-based. A minor shift in data leads to a completely different tree being created [9]. Naive Bayes (NB) and linear discriminant analysis (LDA) are unable to locate a nonlinear structure concealed in high-dimensional results. Secondly, the singularity of inherent matrix is a problem in which the determinant value is zero which leads to nonclassification of matrix [9]. A fuzzy support vector machine (FSVM) was implemented by Nedeljkovic to define and characterize the amount of breast ultrasound [10]. In order to eradicate such errors, algorithms were developed to assist radiologists. Therefore, this distinctive attribute of the tissue patches in the image played an important role in classification. The machine can extract five unique features [11]. Balance them by ADASYN [12] and classification is by multilayer perceptron neural network. The advantage multilayer perceptron neural networks (MLPNNs) MLP is an artificial neural network feedforward architecture that is used to design recognition schemes to identify particular patterns. It is nonparametric learning and is enforceable on a noisy input. It is able to model complex nonlinear and high-dimensional problems. You can pick different kernel functions [9]. Finally, classification is used in the doubtful areas into abnormal or normal detection.

## 2. Related Work

For several years, the community of medical imaging has made attempts to develop CAD framework. With its arrival, novel challenges started emerging, which now require proper knowledge as well as thorough research.

Research has been done on some key modules of CAD. This created a need to develop the computer-aided diagnosis system. It has three aims. First is the detection of the abnormal breast from mammography. The second involves masses' detection, while the third one is meant to differentiate benign from malevolent masses. In this study, the former is focused while it is the essential process of further two attempts. In the previous 10 years, various approaches have been recommended. Milosevic et al. [13] utilized the 20 GLCM features. They used naive Bayes classifier for sorting, keeping up vector machines as well as k-nearest neighbors. Petrosian et al. [14] investigated the utility of texture characteristics for mass and normal tissue classification based on spatial gray-level dependency (SGLD) matrices. Iseri and Oz [15] developed a new method of extraction of features, i.e., statistical analysis based on multiwindow, in order to detect microcalcification clusters. Nababan et al. [16] use three layers of SECoS with 16 features as proposed for classifying benign and malignant masses. Sigh et al. [17] utilized a support vector device that had texture, shape features, and hierarchical technique for categorizing both malignant and compassionate stacks. Perez et al. [18] talked about experimental evaluation and the theoretical description of an innovative attribute collection method that is called uFilter. Via the integrated mammography data as well as MRI, Yang and Li recognized breast cancer. They performed information integration by two techniques, i.e., MIP and TPS. In Kinoshita et al. [19], the mixture of form and texture used provides space for the classification of regular and infected breast lesions based on gray-level cooccurrence matrices (GLCM). Anita and Peter [20] proposed an automated segmentation technique to classify and segment abnormal mass regions on the basis of the maximum cell intensity update. In Peng et al. [21], for initial breast cancer diagnosis in patients with breast microcalcification lesions, FDG-PET/CT was used. Molloi et al. [22] evaluated the breast density through spectral mammography. Kegelmeyer [23] constructed a tool to identify satellite lesions in mammograms and texture characteristics of computed laws from a chart of the local edge orientations. Gorgel et al. [24] suggested spherical wavelet transform. Mohanty et al. [25] recommended a technique that gets ROI by cropping operation. After ROI was extracted, 2D discrete wavelet transform was combined with GLCM in order to obtain texture-based features. There are a total of 65 features that were calculated by this combination. Moreover, PCA was also implemented to eradicate redundant features. At the last step, forest optimization algorithm was implemented to get classification results.

Abdel-Nasser et al. [26] invented technique for change in temperature on normal and abnormal breast cancer detection by extracting GLCM and 22 features and used learning-to-rank and texture analysis methods. Wang et al. [27] developed an algorithm for classifying benign and malignant masses into their appropriate classes. In their work, there were 16 spectrums that contained 16,777,216 features which were further reduced to 18 features by using PCA. The FD was combined with Jaya for training weights and biases of FNN. The projected method was later named Jaya-FNN. Welch et al. [28] did contrast enhancement and also performed dimensioning by CLAHE based adaptive method as well as histogram equalization. The ROI was extracted by using a bimodel processing algorithm in two levels. Firstly, extraction of normal breast boundary was done and then the abnormal breast boundary was extracted. GLCM method was utilized to get the second level statistical texture features. Shape features included eccentricity, LBP, circularity, and Hog. Intensity features included mean kurtoses and skewness. So the feature's space was reduced by a recursive approach. KNN, support vector machine, and decision tree were used for the classification of desirable functions. From the above literature research, segmentation, feature extraction, and feature selection as well as classification are considered as the major factors for categorizing to get better effectiveness of discovery of breast stacks. Mohanty et al. [29] used 19 (GLCM + GLRLM) features of extraction to classify detection of benign and malignant masses. The category imbalance problem [16,30–34] is heavily influenced by machine learning and statistical algorithms. The Heuristic Cover-Sampling Algorithm is a Synthetic Minority Over-sampling Technique (SMOTE). It produces artificial samples from the minority class by parsing existing instances that lie close together. It has been one of the most common methods used for data sample selection for a few weeks [35].

Sampling data approaches are such as Random Over-Sampling (ROS), which replicates extracted features, and Random Under-Sampling (RUS), which removes majority-class samples. In order to adapt to the binary classifier ratio, these methods distort individual counseling [12]. Sampling learning is an active process from datasets through Adaptive Synthetic (ADASYN) algorithm. ADASYN's guiding theory is the use of weighted consideration for the different ethnic groups. The ADASYN approach improves learning in two ways with respect to data distribution: (1) the bias created by the inequality of the class and (2) dynamically altering the boundary of the classification decision to reflect on those samples that are difficult to understand [12].

While each tissue type has its own characteristics for the proposed work, it often hardly differentiates between normal and abnormal cancers. Commonly, cells begin to expand in abnormal cancers and their tissues coloring is visible. Indiscretions have been brought to completion in cell arrays. The cell shows more common in natural tissue and its color is darker. However, there is also a low description of only some low-level dimensions of certain complex systems. In this research, different algorithms were tested to extract features at higher levels on morphological images. So, with extraction algorithms for GLCM features, LBP features, LBGLCM features, GLRLM features, and SFTA features, optimization methods have been attempted in the literature. As an appropriate method to extract features from individual image, each algorithm is applied to the entire dataset.

Unbalancing of dataset, therefore, using hand-crafted features will trigger poor performance from the dataset. The unbalanced data problem is eliminated with the ADASYN algorithm [12], which then deletes irrelevant features by ReliefF that improves training time. Finally, for the classification of data, the feedforward neural network is used.

## 3. Proposed Method

The methodology is adopted to distinguish among eight classes (benign to malignant) according to Breast Imaging-Reporting and Data System (BI-RADS). For such a purpose, preprocessing and segmentation are skipped in this algorithm and restrict the algorithm to four stages, i.e., features extraction, features margin, oversampling, and feature selection and reduction; finally classification is shown in Figure 1.

The model that was mentioned was checked on the INbreast database [36]. For each object, five hand-crafted features (GLCM, GLRLM, LBP, LBGLCM, and SFTA) were extracted from 8 groups of images and their values are stored in a file. For each image, 88 features are obtained by combining these feature vectors. Then, with the ADASYN procedure, the feature vectors of 411 images consisting of 88 functions are oversampled. After this step, 1773 function vectors are generated. Using the ReliefF algorithm, these features were layered down to ten subset functions. In the end, feedforward neural network was modified to multilayer and trained on a selected subset to get a result.

### 3.1. Feature Extraction Method

#### 3.1.1. The Gray Level Cooccurrence Matrix (GLCM)

GLCM is a common method of extraction of texture-based features. By performing an operation in the images due to the second-order statistics, the GLCM decides the textural relationship between pixels. For this procedure, two pixels are normally used [37]. The frequency of variations in these measured pixel brightness values is specified by the GLCM. Namely, it reflects the pixel pairs' frequency creation [38]. As seen in Figure 2, there are several statistical characteristics from a GLCM grey level picture type. The square matrix of features can be denoted by *G* (*i*, *j*). Four distinct forms are used to segment the *G* matrix into regularized typical forming modes. Such patterns are referred to as crossed directions: vertical, lateral, right, and left paths. This can be determined for both neighboring paths.

The Grey Level Cooccurrence Matrix was utilized to extract 22 texture characteristics I-e dissimilarity, association, homogeneity, liveliness dissimilarity, entropy, cluster hue, square variance number, energy, sum variance, sum average, entropy, sum entropy, entropy difference, maximum likelihood, cluster prominence, variance difference, normalized autocorrelation inverse difference moment and measurement details. [39].

#### 3.1.2. Local Binary Pattern (LBP) Feature

A quite effective technique that is responsive to light variations is the extraction algorithm. The LBP method can simply be defined as follows; the image is crossed through a window with a given neighborhood value. And an assignment of an image pixels mark is made. In this step, the threshold is applied according to pixel values adjacent to the middle pixel. The LBP matric is then determined according to clockwise or counter clockwise values in the surrounding neighborhood. Thus, it comprehensively defined the systemic and statistical pattern of the textural system [40]. The LBP algorithm's most key qualities are resistant to changes in the grey level and statistical versatility in real-time applications, which could be used [41].

#### 3.1.3. Local Binary Grey Level Cooccurrence Matrix (LBGLCM)

A combined approach applied along with Local Binary Pattern (LBP) and GLCM is the LBGLCM feature extraction process. The grey level picture is related to the LBP methodology. Instead, since the acquired LBP texture image, GLCM features are removed. At the feature extraction point, the GLCM technique takes adjacent pixels into consideration. It does not execute any procedure in the picture on other local patterns. Textural and spatial knowledge in the picture is collected in accordance with the LBGLCM process. The availability of the LBGLCM algorithm in image processing applications is improved by the simultaneous acquisition of this information [42].

#### 3.1.4. Grey Level Run Length Matrix (GLRLM)

In extracting the spatial properties of gray level pixels, GLRLM uses higher-level statistical techniques. The structure of the features obtained is two-dimensional.

Each value in the matrix reflects the maximum value of the grey level. The characteristics of GLRLM are seven in total. Short-term concentration, long-term focus, and gray-level semi, run-long nonuniformity, take, low gray-level running focus, and overall organization running focus are such high statistical characteristics [43].

(1) $$\begin{array}{c} \text{SRE}=\;\sum_{i=1}^{C}\sum_{j=1}^{R}\frac{P\left(i,j\right)}{j^{2}},\\ \text{LRE}=\overset{G}{\underset{i=1}{\sum }}\overset{R}{\underset{j=1}{\sum }}j^{2}P\left(i,j\right)\;,\\ \text{GLN}={\overset{G}{\underset{i=1}{\sum }}\left[\overset{R}{\underset{j=1}{\sum }}P\left(i,j\right)\right]}^{2},\\ \text{RLN}=\overset{R}{\underset{i=1}{\sum }}{\left[\overset{G}{\underset{j=1}{\sum }}P\left(i,j\right)\right]}^{2}\;,\\ \text{RP}=\frac{1}{n}S,\\ \text{LGRE}=\overset{C}{\underset{i=1}{\sum }}\overset{R}{\underset{j=1}{\sum }}\frac{P\left(i,j\right)}{i^{2}}\;,\\ \text{HLGRE}=\overset{G}{\underset{i=1}{\sum }}\overset{R}{\underset{j=1}{\sum }}i^{2}P\left(i,j\right)\;, \end{array}$$

#### 3.1.5. Segmentation-Based Fractal Texture Analysis

Limited computation time and successful attribute extraction are important in texture analysis. The SFTA solution is a methodology that can be tested in this theory. Throughout the SFTA process, multiple thresholding techniques transform the image into a binary form. Thresholds of *t*1, *t*2, *t*3,…, *tn* are rendered. Interclass and in-class variance values are used to determine the threshold sets. The optimal threshold number is added to the representation regions to minimize the in-class variance value.

Figure 3 demonstrates the extraction steps of the pseudocode SFTA algorithm. The obtained function vector represents VSFTA. Initially, different threshold values (*T*), all pairs of contiguous thresholds (TA), and threshold values (TB) corresponding to the maximum grey level are determined. Then, for all threshold values in the loop, segmented image pixels, boundaries, and VSFTA are modified. The obtained VSFTA vector's asymptotic complexity is *O* (*N*•|*T*|). Although N indicates the number of pixels, |*T*| indicates the number of different thresholds arising from the Otsu multilevel algorithm [44].

### 3.2. Oversampling with Adaptive Synthetic (ADASYN) Algorithm

To address unbalanced class allocation issues for classification activities, the ADAYSN approach is useful. This method is applied to all minority classes. In general, ADASYN bases its operation on weighting the examples of the minority classes according to their difficulty of being learned; therefore more synthetic data will be generated from the more difficult samples, and fewer samples in the case of the easier to learn [12]. This sampling method aims to help the classifier in two ways: first, reducing the error produced by the imbalance of the classes and then focusing the synthetic samples only on the difficult samples to learn [45, 46]. To apply the oversampling method in a multiclass problem, all of the sampled minority classes will be nearer to 1 until the imbalanced rate is nearer to 1. For example, the second is the majority class, with 220 samples, and the first class is with 67 samples; the imbalance rate of these classes is 0.3045. The ADASYN process generates synthetic samples before the rate equal to or nearest to 1 in the method generates 154 samples, generating an imbalanced rate = ∼1.3rd class of 24 samples, the imbalance rate is 0.1090, the method generates 192 samples, the fourth class of 13 samples generates an imbalance rate of 0.05909, and the method generates 209 samples.

In the fifth class of 8 samples, the imbalance rate is 0.0363 and the method generates 208 samples; in the sixth class of 21 samples, the imbalance rate is 0.0954 and the method generates 207 samples; in the seventh class of 50 samples, the imbalance rate is 0.2272 and the method generates 181 samples, and in the last class of 8 samples, the imbalance rate is 0.0363 and the method generates 211 samples of the minority class. ADASY displays the balance of eight groups in Figure 3. The multiple classes' classification problem is described. The algorithm representation is shown in Algorithm 1.

### 3.3. Feature Selection Method

This stage is of significant importance as rarely distinguishable features are discarded, which increases the computational burden on the modeling process. In the present study, ReliefF algorithm was used for dimensional reduction as ReliefF is proved to be computationally efficient and has been proved to be sensitive to complex patterns of association [47–50]. It was used to estimate attributes based upon how their values reflect variations between instances close to each other. By using the abovementioned method, 88 raw features were selected and reduced to 10 optimal features because of their participation topmost according to the weightage to get maximum accuracy. The graph shows 99.5%.

Accuracy at 10 features and 12 features is 100%. This is shown in Figure 4. So that is why we select 10 features. There is not much difference in output, so we skip the remaining ones because that elevates the computational burden of a model. The graph in Figure 4 shows cumulative accuracy against feature numbers which are selected as 10 features that can participate more than total variances.

#### 3.3.1. ReliefF Algorithm

ReliefF is capable of accurately evaluating the quality of attributes with heavy correlations between attributes in classification problems. They have a global perspective by leveraging local knowledge generated by distinct contexts. ReliefF makes a ranking of features according to weight-age and the ones who are participating the most come in the first predictor rank. Other features contain nearly less contribution toward the last as shown in Figure 5. So we can select the 10 most powerful features according to their weight-age and skip irrelevant features that elevate the computational burden of the model [47–49].

Original ReliefF is work done with two classes: difficulties and a stronger class, which deal with noisy data and imperfect data. It is used to calculate feature usability for every feature which can later be applied in order to select features that contain top scores for feature selection. Likewise, ReliefF selects an instance *T* randomly (Step 3), but later, *k* observes the closest neighbors of the same class called the nearest hit values of *H*. So we use the number of nearest neighbors as 3 to mean a positive integer scalar (Step 4), and in the same manner, k-nearest neighbors are the value of one to one of the various classes, called nearest misses *M*(*T*) values (Steps 5 and 6). It also updates the accuracy of the *W*[*A*] class estimate for each attribute *A*, based on their values for *T*, hits *H*, and misses *M*(*T*) (Steps 7 and 8) as in Algorithm 2.

## 4. Classification

### 4.1. Feedforward Neural Network

Classification of morphological images of each class and identifying cancerous conditions seem to be very complex. Feedforward neural network is used to classify tumors [41]. This algorithm is the fastest backpropagation algorithm and is strongly recommended to be used as a first choice supervised algorithm and does not need more memory than others. The network has used four hidden layers. Feedforward neural network was developed by using “newff,” command. The first hidden layer of the network contained 40 neurons having linear transfer function. The second secret layer held 20 hidden neurons. And the third and fourth secret layers contained 10 and 8 hidden neurons. The four-layer network shown (Layer-4) is the output layer and the remaining three layers are hidden layers (Layer-1, 2, 3). The problem under consideration was multilabel classification. For problems with more than two classes, the softmax function is used with multinomial cross-entropy as the cost function; it updated the weight as well as bias values conferring to Levenberg–Marquardt optimization. Data is classified into training, validation, and testing as 60 percent is for preparation, 20 percent is for validation, and the remaining 15 percent is for research. It is fastest for training a moderate-sized FNN. It has been deduced that this optimization is used for approaching second direction training speed without the Hessian matrix. On the other hand, training feedforward networks Hessian matrix can be as

(2) $$\begin{array}{c} H=J^{T}J. \end{array}$$

Gradient will be

(3) $$\begin{array}{c} g=J^{T}e, \end{array}$$

where *J* represents Jacobian matrix having network errors derivate regarding biases and weights and network errors represent vector by “e.” A network has four layers. Each layer has a matrix of “*W*” mass, a vector of ‘b' bias, and an output vector “a.” To differentiate between matrices of weight, vectors of output, etc., in our estimates for each one of these layers, we are adding the layer number as a superscript to the interest variable. In the four-layer network seen in Figure 6, you can see the use of this layer notation and in the calculations at the bottom of the diagram.

The network is shown in Figure 6, below R1 inputs, S1 neurons first layer, S2 neurons second layer, etc. For different layers, it is common to have different neuron numbers. For each neuron, the constant input 1 is fed to the biases.

Notice that each intermediate layer's outputs are the inputs to the following layer. It is also possible to evaluate layer 2 as a one-layer network with S1 inputs, S2 neurons, and a W2 weight matrix of S2 × S1. A1 is the input to layer 2; a2 is the output. Now that we have identified all the vectors and matrices of layer 2 and so on with other layers, the output layer of the network is the last layer. This approach can be adjusting weight as shown in Figure 7.

## 5. Experimental Results and Discussion

The proposed model for MATLAB 2017a has been created. It was used on a Core-i7 processor personal computer with 8GB of RAM as well as 2GB of the graphics card. Mammographic photographs have been used for the study of the scheme proposed. These photographs were taken from the INbreast dataset [26], created by multiple University of Porto institutions, and made available to the public with the permission of the authors. The dataset had a total of 411 images. The matrix of the images was 3328 × 4084 or 2560 × 3328 pixels, while the images were processed in DICOM format. The present research used 411 mammogram images and was further divided into 6 classes according to the Breast Imaging-Reporting and Data System (BI-RADS) class [26] and the classification is shown in Figure 8. It is a risk management and quality assurance method developed by the American College of Radiology that offers a generally recognized lexicon and reporting scheme for breast imaging as shown in Table 1. This refers to mammography, ultrasound, and MRI.

The archive is accessible on this web page.

http://medicalresearch.inescporto.pt/breastresearch/index.php/Get_INbreast_Database.

### 5.1. Performance Analysis of the Proposed Method

Multilabel classification and the closely related problem of multioutput classification are variations of the classification problem where several labels can be applied to each case. Multilabel classification is a generalization of multiclass classification [51], which is the single-label problem of categorizing instances into exactly one of more than two classes; there is no restriction on how many of the classes an instance may be allocated to in the multilabel problem. In our case of Multiclass Classification Issue to be an 8-Class Classification Issue since we have a dataset that has eight class names, sensitivity, precision, and consistency are very critical for the system. Sensitivity reflected the proportion of both positive and genuinely positive events [52]. Specificity showed the percentage of true negative classified cases.

Meanwhile, accuracy depicted the percentage of true positive and true negative correctly classified mammograms. The confusion matrix represented in Figure 8 shows the actual and predicted class count obtained by the classifier. But multiclass classification is an implementation of unlikely binary classification of mammograms. Since the classes here are not positive or negative, at first, it may be a little difficult to find TP, TN, FP, and FN because there are no positive or negative grades, but it is pretty simple. What we did here, for each person class, was to find TP, TN, FP, and FN. We take class BI-RADS 1 and then let us see the values of the metrics from the confusion matrix. Confusion matrix is represented in Figure 8, so we find about true positive (TP) of multiclass values in the diagonal form in green color. If we want to find an overall matrix of TP value, we should add all classes of TP values. For false positive (FP) sum of values in the corresponding column and excluding TP values and for overall, we can sum all classes of FP values. For the false negative (FN) number of values in the following row and except for the TP value, all groups of FN values can be summed overall. For the true negative (TN) class, it is not difficult to take the number of columns and rows and deduct the column and row class. The assessment metrics written below are those of the following.

Sensitivity is used to deal with positive cases only. The ratio of classified to the actual positive cases is shown by sensitivity. When sensitivity is high, the false negative rate is less.

(4) $$\begin{array}{c} \text{sensitivity}=\frac{\text{TP}}{\text{TP}}+\text{FN.} \end{array}$$

Specificity deals with negative cases only. It is used to depict the ratio of actual negative cases to classified ones. When specificity is greater, the false positive rate is less.

(5) $$\begin{array}{c} \text{specificity}=\frac{\text{TN}}{\text{TN}}+\text{FP.} \end{array}$$

Positive predictive value (PPV) is used to deal with positive predictive cases only. The ratio of classified to the actual positive predictive cases is shown by PPV.

(6) $$\begin{array}{c} \text{positive predictive value}\left(\text{PPV}\right)=\frac{\text{TP}}{\left(\text{TP}+\text{FP}\right)}. \end{array}$$

Negative predictive value (NPV) deals with negative predictive cases only. It is used to depict the ratio of actual negative predictive cases to classified ones. When NPV is greater, the false positive predictive rate is less.

(7) $$\begin{array}{c} \text{negative predictive value}\left(\text{NPV}\right)=\frac{\text{TN}}{\left(\text{TN}+\text{FN}\right)}. \end{array}$$

Accuracy deals with the correctness of classification results. The system is considered efficient when accuracy is more.

(8) $$\begin{array}{c} \text{accuracy}=\frac{\text{TP}+\text{TN}}{\text{TP}+\text{FP}+\text{TN}+\text{FN}}. \end{array}$$

Data is classified into training, validation, and testing by using 10 global features, in which 60% is for training, 20% is considered for validation, and the remaining 20% is for testing.

#### 5.1.1. Training on INbreast Dataset

For the training purpose without oversampling, 287 images out of 411 images are used in which 277 images are correctly classified and 10 of them are misclassified. And after using oversampling ADASYN, we used 1241 images out of 1773 images, in which 1233 images are correctly classified and 8 images are misclassified.

#### 5.1.2. Validation on INbreast Dataset

For validation purpose without oversampling, 62 images out of 411 images are used for validation. 60 images are correctly classified for the validation process and 2 are misclassified, and after oversampling ADASYN, 266 images out of 1773 images are used for validation purpose. And all of the 266 images are correctly classified and no image is misclassified.

#### 5.1.3. Testing on INbreast Dataset

For the testing purpose without oversampling, 62 images out of 411 images are used for testing. 59 images are correctly classified testing process and 3 are misclassified class, and after oversampling ADASYN, 266 images out of 1773 images are used for testing purpose, in which 265 images are correctly classified and 1 image is misclassified.

#### 5.1.4. Overall on INbreast Dataset

For the overall talk about without oversampling, 411 images are used in which 396 are correctly classified and 15 images are misclassified.

After applying oversampling ADASYN, 1773 images are used, in which 1764 images are correctly classified and 6 images are misclassified.

### 5.2. Classification Results of Raw Samples

Three phases are included in the proposed framework: feature extraction, feature selection, and classification. Firstly, with 411 samples, the classification results are examined in raw form for 88 features [42]. And then the ReliefF algorithm chooses the 10 most contributory characteristics [50]. Through comparing the output of the classification processes by the FNN algorithm, the contribution of the oversampling system is explored. And there results of each class are shown in Table 2. And individual class accuracy is defined in Figure 9.

Figure 9 shows individual accuracy of each class with samples of classes.

### 5.3. Classification Results Balance by ADASYN

The methods involve four steps: feature extraction, oversampling, feature selection, and classification. Here is the oversampling method ADASYN which helps balance all classes until the imbalanced rate will be closest to 1. And it also prevents overfit problem. ADASYN bases its operation on weighting the examples of the minority classes according to their difficulty of being learned; therefore more synthetic data will be generated from the more difficult samples, and fewer samples are in the case of the easier to learn [25]. The majority class only provides information to quantify the degree of class imbalance, and the number of synthetic data examples to be generated for the minority class in Table 3 shows the output parameters of the 10 most significant feature vectors consisting of 1773 samples of the ADAYSN algorithm. Accuracy of each class is shown in Figure 10. Growing the minority groups with synthetic samples is shown to have a beneficial impact on the accuracy of classification. And the results of each class are shown in Table 3.

The definition made with the inclusion of synthetic samples is seen to generate a contribution of more. One of the most relevant factors is to eliminate the imbalance between classes shown in Table 4. After accuracy level improved, in the confusion matrix, the correctly classified cases are shown in Figure 11. Diagonal is within green color, while misclassified cases are shown in red color. The last column of the confusion matrix shows the sensitivity, precision, and accuracy of the model.

The training state is presented in Figure 12. The gradient is the value of the backpropagation gradient on every iteration. Epoch shows how many iterations should be shown for training purposes. And MU is momentum update which includes weight update expression to avoid the problem of a local minimum.

The performance plot for training is shown in Figure 13. Training mean square error (mse) is downloading which shows perfect training. Best training performance shows few errors determined in Figure 13, which shows 0.0012691 error estimates that are minimal error rate.

The network's ability to estimate the model target is evaluated by showing the regression plot in Figure 14. Regression evaluation can support a model that links between a dependent variable (which you are seeking to forecast) and one or better independent variables (the input of the model). Regression evaluation can determine if there is a considerable link between the independent variables and the dependent variable and the weight of the impact—when the independent variables move, by how much you can predict the dependent variable to proceed. Here we use linear regression to achieve the number of outputs. Linear regression is suitable for dependent variables that are stable and can be fitted with a linear function (straight line). The plot shows that the linear regression of the targets relatively achieves the numbers of outputs.

The plot shows that the linear regression of the training, validation, and testing and overall targets of comparison achieves the number of outputs.

### 5.4. Comparison with Work

Many researchers have worked on those key modules of CAD. This created a need to develop a computer-aided diagnosis system. It has two aims. First is the disclosure of abnormal breasts from mammographic images by an innovative approach. And the second is various classes' classification that uniquely explains all classes according to BI-RADS. For tumor identification, few features contribute to a poor classification due to a slight variation in textures. The present thesis focuses on 5 different algorithms for the extraction of features that can extract different features. Then, because of the overfitting problem, we purpose the oversampling technique by ADASYN that increases the number of samples which also increases algorithm complexity and train time. So for that, we apply feature selection techniques such as ReliefF. And for multiple class classification, we use FNN and the results are shown by a confusion matrix.

Table 5 shows that Abdel-Nasser et al. [2] used local database by extracting 20 optimal features and SVM classifier to obtain accuracy of 88.0%. Pérez et al. [18] in 2011 used DDSM dataset and extracted GLCM + GLCLM 19 features from a region of interest (ROI) to obtain accuracy of 94.9% and furthermore on second hand selected 12 most contribution features of GLCM + GLCLM and got 92.3% accuracy. For classifying tumor region, they used a Boolean vector algorithm. Nababan et al. [16] used Mini MIAS dataset and got 92.26% sensitivity, 92.28% specificity, and 92.27% accuracy. Wang's 16,777,216 features were further reduced to 18 features by using PCA and FFN. Frisk et al. [5] used INbreast dataset and extracting GLCM 16 features from ROI and for classification used SECoS techniques obtaining 82.98% accuracy. Alam and Faruqui [39] expanded the previous work in 2012 and classified by decision tree and obtained accuracy of 96.7% by extracting 19 features and also obtained accuracy of 93.3% by extracting 12 most contributed features. Ozturk et al. used shrunken features which includes GLCM + LBGLCM + GLRLM + SFTA, for oversampling by SMOTE algorithms and classification use and PCA after which they got 94% accuracy for a COVID-19 dataset. We purposed a model by using INbreast dataset; the proposed model focuses on four steps: global feature extraction, oversampling method, feature selection method, and lastly classification and we got 99.5% sensitivity, 99.4% specificity, and 99.5% accuracy.

## 6. Conclusion

Various investigations have been carried out in the field of medicine to study medical disorders and thus to find their correct diagnosis. For this purpose, in the present work, data mining techniques were considered. By utilizing fewer numbers of features, the computational time was reduced without dropping the accuracy of diagnosis. Instead of using complex systems to strengthen the classification accuracy, an effort was made to adopt a simple method to produce a significant result. The results showed 99.5% accuracy which proved the effectiveness as well as the robustness of the proposed system.

## Figures and Tables

**Figure 1:** Methodology of the proposed model.

**Figure 2:** ADASYN oversampling for multiple classes.

**Figure 3:** Pseudocode of SFTA algorithm.

**Figure 4:** Cumulative accuracy against feature numbers.

**Figure 5:** Weight ranking of features.

**Figure 6:** Multiple layers of FNN.

**Figure 7:** Adjusting weight and comparing the output with the target.

**Figure 8:** INbreast dataset of BI-RADS categories.

**Figure 9:** Model shows multiclass samples and obtains each class accuracy.

**Figure 10:** Model shows multiclass samples and obtains each class accuracy by ADASYN.

**Figure 11:** ReliefF optimal features with 1773 samples.

**Figure 12:** Training state of the proposed model.

**Figure 13:** Performance plot showing mse reduction while training.

**Figure 14:** Regression plot for training, testing, and validation.

**Algorithm 1:** ADASYN.

**Algorithm 2:** ReliefF algorithm representation.

**Table 1:** Classification of 8 categories with respective classes.

Breast image categories	Classes	No. of images
BI-RADS 1	Negative	67
BI-RADS 2	Benign	220
BI-RADS 3	Probably benign	24
BI-RADS 4A	Low suspicion for malignancy	13
BI-RADS 4B	Moderate suspicion for malignancy	8
BI-RADS 4C	High suspicion for malignancy	21
BI-RADS 5	Highly suggestive of malignancy	30
BI-RADS 6	Known biopsy-proven malignancy	8

Total	411	

**Table 2:** Classification with raw samples.

Method	ReliefF optimal features with raw samples								
Breast image categories	True positive	True negative	False positive	False negative	Recall rate	Precision	F1-score	Misclassification rate	Accuracy
BI-RADS 1	67	334	0	0	100	100	100	0	100
BI-RADS 2	220	191	0	0	100	100	100	0	100
BI-RADS 3	20	386	1	4	83.3	95.2	88.9	1.2%	98.5
BI-RADS 4A	8	395	3	5	61.5	72.7	66.7	1.9%	98.05
BI-RADS 4B	5	40	2	3	62.5	71.4	66.7	10%	90
BI-RADS 4C	21	382	8	0	100	72.4	84	1.9%	98.05
BI-RADS 5	50	360	1	0	100	98.0	99	0.2%	99.75
BI-RADS 6	5	403	0	3	62.5	100	76.92	0.7%	99.3

**Table 3:** Classification with ADASYN samples.

Method	ReliefF optimal features with ADASYN samples								
Breast image categories	True positive	True negative	False positive	False negative	Recall rate	Precision	F1-score (%)	Misclassification rate	Accuracy
BI-RADS 1	220	1546	0	1	99.5	100	99.8	0.1	99.9
BI-RADS 2	220	1552	1	0	100	99.5	99.8	0.1	99.9
BI-RADS 3	214	1557	0	2	99.1	100	99.5	0.1	99.9
BI-RADS 4A	222	1549	0	0	100	100	100	0	100
BI-RADS 4B	215	1557	0	1	99.5	100	99.8	0.1	99.9
BI-RADS 4C	228	1317	2	0	100	99.1	99.6	0.1	99.9
BI-RADS 5	226	1539	3	5	97.8	98.7	98.3	0.5	99.5
BI-RADS 6	219	1551	3	0	100	98.6	99.3	0.2	99.8

**Table 4:** The comparative results between imbalance and balance samples.

Method	Micro F1 (%)	Macro F1 (%)	Weight F1 (%)	Misclassification rate (%)	Recall rate (%)	Specificity (%)	Precision (%)	Accuracy (%)
ReliefF features with 411 samples	96.35	85.23	96.3	3.54	96.35	98.98	96.35	96.46
ReliefF features with 1773 samples	99.5	99.5	99.5	0.5	99.5	99.4	99.5	99.5

**Table 5:** Result of proposed system and comparison with methodology by using features.

Existing solution	Methodology	Features	Accuracy (%)
Abdel-Nasser et al. [2]	Local database + GLCM + SVM	20	88.0%
Pérez et al. [18]	DDSM + ROI + GLCM + GLCLM + Boolean vector	19 12	94.9% 92.3%
Nababan et al. [16]	Mini MIAS + WFRFT + Jaya-FNN	18	92.27%
Nababan [5]	INbreast + ROI + GLCM + SECoS	16	82.98%
Mohanty et al. [49]	DDSM + ROI + GLCM + GLCLM + decision tree	19 12	96.7% 93.6%
Ozturk et al. [42]	Shrunken features + SMOTE + PCA	20	94.23%
Proposed system	INbreast + (GLCM, LBP, LBGLCM, GLRLM, and SFTA) + ADASYN + FNN	10	99.5%

## Data Availability

The archive is accessible on the web page http://medicalresearch.inescporto.pt/breastresearch/index.php/Get_INbreast_Database.
